The article "Construction and Model Realization of Financial Intelligence System Based on Multisource Information Feature Mining" was published in 2022. Journal: Comput Intell Neurosci.

# Construction and Model Realization of Financial Intelligence System Based on Multisource Information Feature Mining

**DOI:** 10.1155/2022/9363023

**Published:** 2022-07-04

**Authors:** Jing Li

**Affiliations:** School of Henan Institute of Economics and Trade, Zhengzhou 450000, Henan, China

## Abstract

Multisource information mining systems and related business intelligence technology are currently a hot topic of research. However, the current commercial applications and applications are not ideal in terms of application. Because there is still much work to be done before decision support, it is best to transition to them only financially. This paper examines the multisource part of the information used in mining and introduces research hotspots in the fields of accounting informatization, the development status of intelligent financial analysis software, the research and application status of data warehouse, data mining, and decision support systems. This paper examines the specific composition and content of a financial information system using information mining to lay a solid foundation. Financial intelligent analysis, financial intelligent monitoring, financial intelligent decision-making, and financial intelligent early warning are the four parts of the financial intelligent system. It then examined the structure and processing of the financial intelligence system and proposed a financial intelligence system operation strategy. Financial intelligence low-risk integrated implementation strategies and ideal financial intelligence models, according to the current state of research and practical applications. According to the findings, the overall discrimination accuracy of the financial information system based on mining multisource information features is up to 95%, which is 42% higher than the traditional model. The development and use of financial information benefit from the realization and exploration of the financial intelligence system model.

## 1. Introduction

Industrialization, processization, and decision-making are the three stages of the development of an information system. Financial records can neither fully reflect the work level and needs of modern network technology and enterprise records nor they fully cover their important content, due to the rapid development of network information technology. Communication will consider not only the use of information technology but also its financial impact on the company. It differs from traditional records and computer people who are only interested in technology or dealing with a specific machine component. A financial decision support system (FDSS) is a computer-assisted decision-making process that assists industry –decision makers in obtaining relevant data. Small-scale processing and financial management models, for example, have a relatively poor financial status in terms of economic management. Intelligent financial systems are popularizing China's accounting information system at the same time. The system's benefit is that it can display and provide information about business efficiency. ERP business management software also has a business intelligence application. From a difficult decision to a scientific one, the decision-making process has evolved. Financial information, sales information, purchasing information, and production information are all covered by business intelligence, which brings financial business information to the world of financial software. Financial information includes the ability to identify short-term solutions to complex problems, the ability to test the impact of various strategies, the ability to test new ideas and insights, good management skills, low costs, and the ability to make objective and important decisions. The audit and execution of financial information will become the focus of financial statement auditing and execution under the guidance of this system.

The article "Construction and Model Realization of Financial Intelligence System Based on Multisource Information Feature Mining" was published in 2022. Journal: Comput Intell Neurosci.

As an important branch of data analysis in the computer field, machine learning mainly analyzes data, mines potential laws, and uses laws to predict unknown samples, that is, to discover and count useful information, knowledge, and even wisdom from data. As an interdisciplinary field, machine learning mainly includes ensemble learning, semisupervised learning, transfer learning, and rule learning. Among them, rule learning, as a research method of knowledge discovery in the field of machine learning, mines hidden patterns or rules with practical significance from data. For classification problems, rule learning is often used to make judgments about the class labels of unknown samples. Classification-oriented rule learning methods have been widely used in various practical application fields. For example, in the structural information prediction of biological proteins, the function of protein structure can be predicted by using rule learning. In judging the type of mechanical failure, it is possible to determine what kind of failure the machine has by learning the rules. This paper uses the method of multisource information mining features to design and implement the construction of financial function system.

First, research the inevitable development process required to support future computing, financial intelligence, with specific and long-term goals in mind, such as creating a platform for account computing and business intelligence, as well as ample space for follow-up. Second, it is through the promotion and implementation of intelligent financial analysis systems, such as cabin management, electronic reporting, and clear tables, which is exactly what is required for statistics and is also a key factor for accountants that education will gradually transform. Third, from the standpoint of businesses, research ideas guide the employment transformation of financial practitioners while also using computers to collaborate, so that financial practitioners can lead financial practitioners into the information age.

The article "Construction and Model Realization of Financial Intelligence System Based on Multisource Information Feature Mining" was published in 2022. Journal: Comput Intell Neurosci.

## 2. Related Work

In the construction and realization of the financial intelligence system, many experts at home and abroad have done the research. Zhang W believed that the intelligent financial system can improve the utilization rate of data, improve the work efficiency of financial personnel, and increase the security of financial processing services. The system can help managers make important financial decisions, financial budgets, etc. [1]. *D* Aikman et al. provided a framework for assessing the accumulation of vulnerabilities in the financial system. They collected 46 indicators of financial and balance sheet health, covering valuation pressures, nonfinancial borrowing, and measures of financial sector health [2]. Prochniak M et al.'s study aimed to analyze the impact of the development and stabilization of the financial sector on economic growth based on quantitative methods that yield robust results. It is tested that the relationship between the development of the financial sector and economic growth is nonlinear [3]. Polzin F et al. believed that diversification makes financial systems more resilient. Furthermore, the transition to a more sustainable energy system presents diverse financial investment needs [4].

However, the traditional financial system construction is not perfect, and there are many shortcomings, so in the experiment, the paper uses the method of multisource information feature mining to construct the functional financial system. Han *Z* et al. proposed a method to identify key assembly structures in assembly models from the perspective of assembly topology and multisource properties. The assembly model is based on complex network representation, and a two-level evaluation model is proposed to evaluate the importance of assembly parts [5]. *X* Gao et al. believed that the Dempster–Shafer theory has inestimable value in dealing with uncertainties in the field of multisource information fusion, but how to fuse highly conflicting information is still an open question [6]. Wu B et al.'s research proposed a multisource information fusion method combining cloud model, support vector machine, and evidence-based reasoning. In the data processing stage, various information sources are trained through different models to analyze financial value at risk [7]. Wu Y et al. believed that the multisource information fusion model consists of three heterogeneous meta-learning machines, namely, neural network, support vector machine, and random forest, and the final metaspectrum can be obtained by executing the final decision method [8]. However, the above data have not been recognized by the public because the experimental process is not rigorous enough.

The article "Construction and Model Realization of Financial Intelligence System Based on Multisource Information Feature Mining" was published in 2022. Journal: Comput Intell Neurosci.

## 3. Multisource Data Mining Source Ensemble Learning Method

In reality, many application fields [9, 10] are faced with multisource data sources, and the structure information of data sources is inconsistent; that is, data sources are divided into two categories: labeled data sources and unlabeled data sources. Therefore, it is difficult to traditionally integrate multiple data sources directly into a single data source for learning. Based on this, the research makes full use of the label information of the labeled data source and the internal structure information of the unlabeled data source, proposes two label propagation methods to make the unlabeled data source have class labels, and then constructs an ensemble learning method of multiple data sources. The experimental results showed that compared with the two traditional classification algorithms [11], the multiheterogeneous data source ensemble learning method based on label propagation has higher classification accuracy, better robustness, and stronger scalability. In addition, when the number of unlabeled data sources is large, the local consistent label propagation method is better than the global consistent label propagation method.

Multisource data source ensemble learning is essentially a multiclassifier system in which subclassifiers are trained by local data sources.  Figure 1 shows the integrated learning framework of multisource data sources. The main ideas are given as multiple data sources; based on label propagation to make unlabeled data sources have labels, a base classifier is obtained by training each local data source, and the result pair distribution of the multibase classifier is fused, which tests the classification results of samples in different data sources as the final prediction results. Based on the ensemble learning framework for obtaining multisource data sources, the following will introduce the two label propagation methods of global consistency and local consistency in detail and point out that these two label propagation methods are mutually replaceable.

The research provides a multisource information system composed of multiple data sources. First, the sampling range is computed at each local data source to obtain a set of local decision rules [12]. Second, the rules are constrained by certain local decision-making standards; local decision-making standards that do not meet the minimum coverage are removed, and selection is made according to the minimum coverage. Third, the votes for each rule are counted in all local decision documents, and some rules for candidate decision voting include the global coverage and global average coverage of candidate decision rules [13]. Finally, the decision rules that do not meet the world average are excluded from the decision-making rules set by the high-voted candidates, and all the decision-making rules that get high votes are combined. The specific algorithm flow is shown in Figure 2.

The article "Construction and Model Realization of Financial Intelligence System Based on Multisource Information Feature Mining" was published in 2022. Journal: Comput Intell Neurosci.

### 3.1. Using Weights to Synthesize Decision Rules

Given a multisource decision information system, neighborhood granulation is used to extract decision rules from each local data source, and these decision rules are, respectively, forwarded to the corresponding knowledge base. Meanwhile, the decision rules in the knowledge base are called local decision rules. Finally, all local decision rules are synthesized to solve the global decision rules [14]. In order to synthesize global decision rules from multiple knowledge bases, the weight of each data source is obtained by learning, and the weight is used to infer the neighborhood size of each global decision rule.  Figure 3 presents the framework of a multisource decision rule synthesis model [15]. The traditional multidata source learning algorithm concentrates the data from all data sources into a unified data source for processing, which will lead to problems such as large data volume, data privacy leakage, and high transmission cost. Compared with traditional methods, the method using the weight synthesis model can effectively avoid these problems, thus providing a new feasible technique for multi-information source knowledge discovery [16].

### 3.2. Integration Model

Different data sources can provide descriptive information from different perspectives of the sample set, so the integrated learning model can be built directly on the multisource information system. To build an ensemble model on multiple heterogeneous data sources, on the basis of label propagation through global consistency or local consistency, all data sources describing the training sample set have class labels [17]. Among them, Figure 4 shows the label propagation algorithm based on global consensus.

### 3.3. Dataset and Its Statistics

This study introduces two real-world datasets used to evaluate recommendation performance, including their preprocessing and simple statistics on the datasets. Then, the evaluation metrics and evaluation protocol of recommendation performance are given. It is evaluated on two datasets: Epinions and Ciao [18]. Users can rate items, trust relationships can be established between users, and users can express their opinions on products and write review texts. First, it needs to eliminate stop words, and then, select the first *L* = 8000 words by word frequency as vocabulary. To reduce noise and errors, it keeps only users who clicked on at least 4 items and deletes those users with only 1 or 2 points [19]. The item index in the rating matrix corresponds to the document index of the document matrix in the review repository, that is, combining all user reviews of an item into the total reviews of an item [20]. The final statistics are shown in Table 1.

The article "Construction and Model Realization of Financial Intelligence System Based on Multisource Information Feature Mining" was published in 2022. Journal: Comput Intell Neurosci.

It can be found that the scores on both datasets are very sparse, and the average length of documents on the Epinions dataset is very short. The average number of comment words contained in each item on the Ciao dataset is 42 times that of Epinions, and Ciao's social relationship density is 12 times that of Epinions. Therefore, the additional data sources are included in the Ciao dataset; information reviews and social information are richer and of higher quality, and they can be expected to have a greater impact on the final recommendation performance. This observation is consistent with previously obtained quantitative assessments. A more compact use of scoring information and social information, that is, capturing social influence with a neighbor graph structure through trust values, can improve the RMSE prediction performance on both datasets. For example, compared to the LOCABAL model, the eSMF model has a relative RMSE performance improvement of 1.18%, 0.89%, and 0.72% when the Epinions training set accounts for 20%, 50%, and 70%, respectively, as shown in Figure 5.

### 3.4. Evaluating the Multisource Information Fusion Model

Mean: this method uses the mean of the scores in the entire training set to predict, which is the term *μ* in the formula. This method is the best constant prediction under the RMSE metric [21]:

(1) $$\begin{array}{c} {\overset{⌢}{R}}_{u,i}=\mu +b_{u}+b_{i}+P_{u}^{T}Q_{i}. \end{array}$$

In this method, PMF decomposes the scoring matrix to learn user and item feature vectors, as shown in the formula. It is a representative method of hidden factor collaborative filtering, which only utilizes the scoring data source:

(2) $$\begin{array}{c} \underset{P,Q}{\min}{\sum_{Ru,i\neq 0}\left(R_{u,i}-{\hat{R}}_{u,i}\right)}^{2}+\lambda \left({\left\|P\right\|}_{F}^{2}+{\left\|Q\right\|}_{F}^{2}\right). \end{array}$$

The LOCABAL method is based on matrix factorization, exploiting both social local and global context, as shown in Equations 3–6. It is a representative method of the social matrix decomposition method, which only utilizes the scoring data source and social information:

(3) $$\begin{array}{c} \underset{P,Q,H}{\min}\sum_{Ru,i=0}\left(R_{u,i}-{\hat{R}}_{u,i}\right), \end{array}$$

(4) $$\begin{array}{c} \lambda_{rel}{\sum_{T_{u,u\neq 0}}\left(S_{u,v}-P_{u}^{T}HP_{v}\right)}^{2}+\lambda_{\text{norm}}\Omega \left(\Theta \right). \end{array}$$

HFT hidden topics are learned from reviews, as shown in the formula. It is a representative method of the topic matrix factorization method, which only utilizes the scoring data source and comment text information. The RMSE comparison results are shown in Table 2.

(5) $$\begin{array}{c} \underset{P,Q,\Phi }{\min}\sum_{Ru,i\neq 0}{\left(R_{u,i}-{\hat{R}}_{u,i}\right)}^{2}, \end{array}$$

(6) $$\begin{array}{c} \lambda_{rev}\sum_{d-1}^{N}\sum_{n\in Nd}\left(\log\;\theta_{z\;d,n}+\log\;\varphi_{z\;d,n,w\;d,n}\right). \end{array}$$

The data have shown that eliminating all auxiliary data sources MR3/content/social from the fusion model MR3 results in a 7.99% decrease in the overall relative RMSE, and the study wanted to know how the additional data sources helped the MR3 model improve its predictive performance. The problem can be examined from the richness of review data and social information.  Figure 6 shows the prediction performance of MR3 and its S components.

The article "Construction and Model Realization of Financial Intelligence System Based on Multisource Information Feature Mining" was published in 2022. Journal: Comput Intell Neurosci.

For the first time, this paper proposes the MR3 fusion model, which can use multiple recommendation data sources at the same time. Unlike other fusion models, both components used are tried and true techniques. Simultaneously, an efficient extended social recommendation model, eSMR, is obtained, and the efficiency of the two proposed models has been verified on two large-scale datasets, indicating that recommendation performance can be improved further by using the neighbor graph structure and adding additional data sources. We will discuss how to extend the fusion model MR3, which mines implicit feedback information from scoring data sources, in order to delve deeper into the limited recommendation data sources. The fusion model and the extended fusion model both mine implicit feedback, and their model parameter learning processes are similar.  Figure 7 shows the multisource information mining performance prediction.

### 3.5. Evaluation and Selection Methods of Information Source Quality

Multi-information sources refer to providing description information from multiple perspectives for the same sample set. First of all, it is pointed out that importance and redundancy are two important factors for evaluating the quality of information sources. Among them, the degree of importance represents the contribution of one information source to the classification, and the degree of redundancy represents the degree of overlap of the available information in different information sources. Second, a metric is devised using mutual-neighborhood information to assess quality and select information sources with the highest importance and least redundancy. Experimental results show that the metric is useful for finding a range of task-relevant information sources and outperforms many commonly used methods. Given a random variable, the entropy of A is defined as follows:

(7) $$\begin{array}{c} H\left(A\right)=-\sum_{i=1}^{n}p\left(a_{i}\right)\log\left(a_{i}\right), \end{array}$$

(8) $$\begin{array}{c} H\left(A,B\right)=-\sum_{i=1}^{n}\sum_{j=1}^{m}p\left(a_{i},b_{j}\right)\log\;p\left(a_{i},b_{j}\right), \end{array}$$

(9) HA|B=HA,B−HB=−∑i=1n∑i=1mpa,ibjlog  pai|bj.

The article "Construction and Model Realization of Financial Intelligence System Based on Multisource Information Feature Mining" was published in 2022. Journal: Comput Intell Neurosci.

Given A and B, the mutual information between A and B is

(10) $$\begin{array}{c} MI\left(A;B\right)=-\sum_{i=1}^{n}\sum_{j=1}^{m}p\left(a_{i},b_{j}\right)\log\frac{p\left(a_{i}|b_{j}\right)}{p\left(b_{j}\right)}. \end{array}$$

To describe the numerical or discrete feature set F, the neighborhood of sample *x* on *f* is defined as f(x), so the uncertainty of the example in this field is defined as follows:

(11) $$\begin{array}{c} NH_{xi}^{\delta }=-\log\frac{\left\|\delta_{f}\left(x_{i}\right)\right\|}{n}, \end{array}$$

(12) $$\begin{array}{c} NH^{\delta }\left(f\right)=-\frac{1}{n}\sum_{i=1}^{n}\log\frac{\left\|\delta_{f}\left(x_{i}\right)\right\|}{n}. \end{array}$$

Suppose *r* and *f* are two self-feature sets. The conditional neighborhood entropy of *r* with respect to *f* can be defined as follows:

(13) $$\begin{array}{c} NH^{\delta }\left(r,f\right)=-\frac{1}{n}\sum_{i=1}^{n}\log\frac{\left\|\delta_{f\cup r}\left(x_{i}\right)\right\|}{n}, \end{array}$$

(14) $$\begin{array}{c} NH^{\delta }\left(r,c\right)=-\frac{1}{n}\sum_{i=1}^{n}\log\frac{\left\|\delta_{r\cup c}\left(x_{i}\right)\right\|}{n}, \end{array}$$

(15) $$\begin{array}{c} NH^{\delta }\left(r|f\right)=-\frac{1}{n}\sum_{i=1}^{n}\log\frac{\left\|\delta_{r\cup f}\left(x_{i}\right)\right\|}{\left\|\delta_{f}\left(x_{i}\right)\right\|}, \end{array}$$

(16) $$\begin{array}{c} NMI^{\delta }\left(r;f\right)=-\frac{1}{n}\sum_{i=1}^{n}\log\frac{\left\|\delta_{r}\left(x_{i}\right)\right\|•\left\|\delta_{f}\left(x_{i}\right)\right\|}{n\left\|\delta_{r\cup f}\left(x_{i}\right)\right\|}. \end{array}$$

In the process of information source selection in a multisource environment, a set of information sources with the greatest contribution to the classification is selected first. Usually, the selection process of information sources is based on the magnitude of importance. Therefore, the formula for selecting according to the importance of the information source is

(17) $$\begin{array}{c} SU\left(f_{1};f_{2}\right)=2\left[\frac{MI\left(f_{1};f_{2}\right)}{H\left(f_{1}\right)+H\left(f_{2}\right)}\right], \end{array}$$

(18) $$\begin{array}{c} NSU^{\delta }\left(f_{1};f_{2}\right)=2\left[\frac{NMI^{\delta }\left(f_{1};f_{2}\right)}{H^{\delta }\left(f_{1}\right)+H^{\delta }\left(f_{2}\right)}\right], \end{array}$$

(19) $$\begin{array}{c} TSU^{\delta }\left(F;c\right)=\frac{nNSU_{cf}^{\delta }}{\sqrt{n+n\left(n-1\right)NSU_{ff}^{\delta }}}, \end{array}$$

(20) $$\begin{array}{c} \max\;D\left(S,c\right),D=\frac{1}{\left|S\right|}\sum_{si,\notin S}TSU^{\delta }\left(s_{i};c\right). \end{array}$$

In addition, ten-fold cross-validation method and ensemble learning based on majority voting are used to verify the classification ability of the proposed algorithm; that is, for each dataset, one hundred information sources are generated ten times, and ensemble learning is performed based on multiple information sources each time to obtain classification accuracy. Then, the average of the ten running results is used as the final classification accuracy. In addition, the threshold of the neighborhood is set to 0.01 and the class label of each information source is consistent with the class label of the original dataset, as shown in Table 3.

The article "Construction and Model Realization of Financial Intelligence System Based on Multisource Information Feature Mining" was published in 2022. Journal: Comput Intell Neurosci.

## 4. Financial Intelligence System Architecture and Implementation Strategy

The overall architecture of the financial intelligence system is divided into three layers, the data acquisition layer, the data organization storage organization layer, and the data analysis display layer, as shown in Figure 8.

Data are extracted from the original business processing system by the data acquisition layer. Internal financial system, internal accounting management system, local external financial system, remote external financial system, and so on are all included. The financial data are loaded into the data warehouse, and the material data are prepared for the construction of the next analysis model, thanks to data extraction, cleaning, conversion processing, and comprehensive improvement. The data organization and storage layer, which includes the data warehouse, is a platform for organizing and storing data retrieved from the data source after ETL. ETL tools are used to extract, clean, update, process, and synthesize source data to create a comprehensive statistical element library. The data layer of each granularity is an enterprise-level global data repository established according to the needs of subject analysis, and it includes detailed level, light integration level, medium level, and high level integration. Because the data warehouse is different from a traditional database, its management is also different. The data warehouse serves as the foundation for the method base, model base, knowledge base, and multidimensional analysis model base. The method library provides data mining and data analysis method guidance. Concrete models are available in the model library. The knowledge base converts data and information into knowledge by processing the results of data mining and data analysis. The purpose of the multidimensional analysis model library is to keep a hierarchical analysis model of commonly used dimensions and to answer complex analysis questions quickly. Multidimensional reporting, multidimensional analysis, and data mining tools, as well as interactive imaging and data drilling technology, are used in the data analysis display layer. All tasks such as reporting, analysis, and charting can be done quickly and easily in a relaxed environment, enhancing the data volume and providing truly informative data.

The article "Construction and Model Realization of Financial Intelligence System Based on Multisource Information Feature Mining" was published in 2022. Journal: Comput Intell Neurosci.

### 4.1. Advantages of Low-Risk Financial Intelligence Implementation Strategies

ERP is a “top-level project,” and the financial intelligence mainly used for decision support for senior managers is data engineering. The support of senior managers is directly related to the success or failure of implementation. The traditional financial intelligence implementation strategy has long battle lines, and the establishment of data warehouses is difficult. The main reason is that data warehouses are subject-oriented, and managers have an insufficient understanding of requirements. In addition, today's social environment changes very fast, so the themes often change, which makes it very difficult to implement and extend the front line, and a lot of resources are invested but no effect can be seen. If the data cannot see the effect, it will not support the implementation of the project, and the lack of data to support the project will make it more difficult to implement and even directly lead to the failure of the project implementation. The adoption of low-risk financial intelligence strategies can allow managers to see the visual display and analysis of data for decision support through some simplified processes from time to time and constantly communicate with managers to understand their needs in the process. Through the continuous promotion of the low-risk implementation strategy, the managers' understanding of the entire system has been continuously improved, and the requirements put forward on this basis are more targeted and reasonable. In this way, the confidence in the implementation of financial intelligence will be enhanced, the support of data will be obtained, and the probability of successful project implementation will be greatly improved.

The article "Construction and Model Realization of Financial Intelligence System Based on Multisource Information Feature Mining" was published in 2022. Journal: Comput Intell Neurosci.

In the implementation of the financial intelligence system, the business personnel should be the protagonists compared with the technical personnel. The business personnel should make detailed analysis on the macro demands put forward by the decision makers, and the technical personnel should provide the platform and technical support for the business personnel. In the low-risk financial intelligence implementation strategy, through simple training of business personnel, they can turn data into information, visualize and interactively display it, improve business insight, and discover knowledge from information.  Table 4 is the data structure of the voucher and detailed table.

### 4.2. Low-Risk Financial Intelligence Implementation Strategy Practice

From the above analysis, it can be seen that using ExcelCrystal and EasyTable tools, we can realize data warehouse, data mining, OLAP, interactive data, visualization data analysis, and other functions. From the perspective of business personnel, these two programs do not require programming or coding. After self-study or simple training, they can create excellent interactive visualizations according to their own business. Excel is a common data analysis software used by any enterprise. As long as you have a little understanding of the business, it is a boon for those who simplify the business. The training bit can master the skills of data mining and analysis. Therefore, at this stage, management decisions can be fully supported by implementing a low-risk financial intelligence strategy. Here is an example of data drilling in a sales report, showing how to achieve low-risk financial intelligence through the combination of Excel and Crystal Xcelsius. Sales data are generally the basis for the analysis and evaluation of business performance, but sales data are generally very large, with many dimensions, and there are many levels under each dimension. Faced with a large amount of complex data, in the past, when managers needed data, they needed to filter and summarize these large amounts of data to obtain the required data of the corresponding dimensions and levels. However, when the demand changes and other information is needed, these large and complex data must be filtered and summarized to obtain data of other dimensions and levels. These tasks will be repeated every time the requirements change, and different reports will be provided. The timeliness and accuracy of the reports are very low, which seriously affects the decision-making. And EXCEL's pivot table summarizes all the data into a pivot table and then sets multiple page fields such as year, region, product category, price, and channel to realize the multidimensional display of data, as shown in Table 5.

The article "Construction and Model Realization of Financial Intelligence System Based on Multisource Information Feature Mining" was published in 2022. Journal: Comput Intell Neurosci.

Due to the flexibility of the pivot table, each field can be dragged and placed at the desired position, and many data can be constructed into multidimensional tables to display all the data, and then filter out the required data. It can be seen that the more page fields are set, the more data can be stored. Not only page fields but also row fields and column fields can be added to increase the dimension of data. And it is also very flexible in the processing of time, which can be aggregated by month, quarter, year, and even by hour, minute, and second. In this way, when the management requirements change, the required data can be found by simply dragging and dropping, and the information needed for decision-making can be obtained quickly and accurately. In addition, a chart analysis model with analysis and graphic display functions can also be drawn, as shown in Figure 9.

Product sales revenue is the key monitoring of enterprises. In this model, the line chart on the right can easily monitor the actual sales and planned sales amount of each product each month and the forecasted sales for future months based on that. The difference between actual and planned is visualized by the scale on the left. The scale at the bottom left shows the sales contribution of each product in the form of a pointer. In the upper right bar area, you can monitor the cumulative actual sales, planned cumulative sales, and corresponding variances for each product.  Figure 10 is a comparison of financial system performance between traditional financial statistics and multisource information feature mining.

## 5. Discussion

In this model, there are not only two variables of sales volume and adjustment volume but also intuitive understanding of the value of income. The model uses a structure diagram to illustrate the relationship between several factors that affect profitability. For example, by setting the variable cost sliders, change the different factors that affect changes in value, total cost, and final revenue. The revenue growth model uses a transition line with advance notice. If the profit is positive, the growth line will appear green, and if the profit is negative, the loss line will appear red, creating a red flag and attracting the attention of decision makers. In the transaction progress process, there is an initial alert table that visually determines the gap between current transaction volume and downtime and provides a way to adjust the gap. Also, for breakeven, you can change unit prices, fixed or variable prices, change breakeven sales, etc.

The article "Construction and Model Realization of Financial Intelligence System Based on Multisource Information Feature Mining" was published in 2022. Journal: Comput Intell Neurosci.

Furthermore, the model includes an operational risk dashboard that allows decision makers to see the impact of various factors on profits in their current state. When the selected factors move in an unfavorable direction in the current state, operational risk is defined as the percentage impact on profits. To select the influencing factors, click the “factor selection” button and then choose the single most important influencing factor. Check “unit price” to see the impact of unit price changes on profit; if the sales volume is unstable, check “sales” to see the impact of sales volume changes on profit, etc., that is, single factor analysis. It can also be chosen multiple important factors, such as unstable product prices and unstable raw material supply prices; simply check “unit price” and “material” to see how these two factors interact to affect profits, which is known as multifactor analysis. The business subinsurance is displayed as a dashboard, and an early warning system is used to visually see the impact of the selected factors on profit in the current state. There are also scheme buttons in this model for saving, loading, and deleting schemes, allowing users to save their results after adjusting all of the variables, as well as view and delete them after loading.

## 6. Conclusion

Financial data are primarily used for business management decision-making, and Chinese SMEs are limited in their use and promotion of financial data due to a variety of factors including capital and technology. Financial intelligence solutions that are both cost-effective and simple to use are in high demand. On the basis of research on some of the financial intelligence products currently used by large domestic enterprises, this paper examines the basic theories of business intelligence and financial intelligence, as well as the construction of financial intelligence in small- and medium-sized enterprises. The following are the main aspects of this paper's research findings: propose a low-risk enterprise financial intelligence strategy and locate the enterprise financial information system model construction. This is the conclusion reached after examining existing technical abilities and previous knowledge, as well as the characteristics of EXCEL and Xcelsius. An example of financial intelligence analysis, an example of financial intelligence monitoring, an example of financial intelligence decision-making, and an example of financial intelligence early warning are all established on the basis of the actual combat financial system. These examples enable businesses to assess the feasibility of the proposed financial intelligence application scheme. The use of multisource information feature mining and VBA technology in EXCEL in the technical realization is the most notable feature of this paper's research results. Their use among Chinese financial personnel is rapidly spreading due to their outstanding performance. Because the design and construction of a financial intelligence system is a very complex project, only a few parts that are closely related to the research of this topic are included in this paper, as well as some issues that have not been discussed, due to time, materials, and the author's own ability. This paper only provides a broad classification of financial intelligence systems and attempts to implement some common models. It is also necessary to conduct extensive research on the specific models of each component, which is a continuous improvement process. In the realization of financial intelligence, this paper mainly not only considers adopting low-risk financial intelligence implementation strategies but also needs to do in-depth research on ideal and comprehensive implementation strategies. This research focuses on financial intelligence, but after the research and application of financial intelligence are fully mature, it is necessary to study the transition to business intelligence and even decision support on this basis.

The article "Construction and Model Realization of Financial Intelligence System Based on Multisource Information Feature Mining" was published in 2022. Journal: Comput Intell Neurosci.

## Figures and Tables

**Figure 1:** An ensemble learning framework for multisource data sources.

**Figure 2:** The mining process of high-voting decision rules in multisource information systems.

**Figure 3:** Decision rule synthesis model in multisource information system.

**Figure 4:** ELMG algorithm framework.

**Figure 5:** Comparison of the eSMF model with a standard social matrix decomposition model LOCABAL.

**Figure 6:** Prediction performance of fusion model MR3 and its S components.

**Figure 7:** Prediction performance of fusion model MR3.

**Figure 8:** Financial intelligence system.

**Figure 9:** Graphical presentation model of sales data.

**Figure 10:** Product sales revenue monitoring.

**Table 1:** Dataset statistics.

Statistics	Epinions	Ciao	Notes
User number	49454	7340	56794
Number of items	74154	22472	96626
Ratings/comments	790940	183947	974914
Social relationship	434680	112942	547622
Word count	2246837	288740000	31120837
Scoring density	0.00022	0.0011	N/A
Social density	0.00018	0.0021	N/A
Average number of words per item	30.3	1284.9	N/A
Average number of relationships per user	8.78	15.38	N/A

The article "Construction and Model Realization of Financial Intelligence System Based on Multisource Information Feature Mining" was published in 2022. Journal: Comput Intell Neurosci.

**Table 2:** RMSE comparison of fusion model MR3 and different methods.

Datasets	Training (%)	Methods				
		Mean	PMF	HFT	LOCABAL	MR3
Epinions	20	1.2265	1.2001	1.1857	1.1222	1.1051
	50	1.2239	1.1604	1.1323	1.1055	1.0809
	80	1.2225	1.1502	1.0960	1.0892	1.0648
	90	1.2187	1.1484	1.0867	1.0840	1.0634

Ciao	20	1.1095	1.0877	1.0439	1.0287	1.0142
	50	1.0964	1.0536	1.0379	0.9930	0.9740
	80	1.0899	1.0418	0.9958	0.9709	0.9521
	90	1.0841	1.0391	0.9644	0.9587	0.9451
Average						

**Table 3:** Descriptive information for the dataset [22].

Datasets	Samples	Features	Classes
COLON	62	2000	2
SRBCT	63	2308	4
TOX-171	171	5748	4
PIE10P	210	2420	10
AR10P	130	2400	10
YALE	165	1024	15

**Table 4:** Data for the voucher schedule.

Serial number	Field name	Illustrate	Type	Length
1	I-id	Unique ID when entering	Int	4
2	I period	0 refers to the initial transaction detailed account, 21 refers to the preliminary bank account to be checked, 20 refers to the balance before adjustment of the bank account, and 1 refers to the voucher and details	Tinyint	1
3	Csign		Varchar	8
4	I signseq	According to the assignment by the system, it can be null at the beginning of the period	Int	4
5	Ino-id	The voucher number is assigned by the system and can be null at the beginning of the period	Smalint	2
6	Inid	Assigned by the system, it is 1 at the beginning of the period	Smalint	2
7	Dbill-date	Amendments to a limited range of dates available	Datetime	8
8	Idoc		Smalint	2
9	Cbill		Varchar	20
10	Ccheck		Varchar	20
11	Cbook		Tinyint	20
12	IBook		Varchar	1
13	Ccashier		Varchar	20
14	Iflag		Tinyint	1
15	Ctex1		Varchar	10
16	Ctex2		Varchar	10
17	Cdigest		Varchar	60
18	Ccode		Varchar	15
19	Cexch-name		Varchar	8

**Table 5:** Pivot table analysis model for sales data.

Year	Date	Children's products	Clothing	Food	Sporting goods	Artwork	Bike
2019	Season 1		68		336	805	685
	Season 2	63	5372	1166		1969	1204
	Season 3	182	2825	2734	341	1752	1294
	Season 4		8232	2215		855	1533

2020	Season 1	194		304	375	1134	
	Season 2		3458	1192	229	800	1285
	Season 3	203	6756	2680	961	1350	1670
	Season 4	103					

2021	Season 1		5555			940	2824
	Season 2	255	4076	3100	279		
	Season 3		7945		551	2192	2557
	Season 4	235					

## Data Availability

The data used to support the findings of this study are available from the author upon request.
